The article "Parameter estimation of the Solow–Swan fundamental differential equation" was published in 2022. Journal: Heliyon.

# Parameter estimation of the Solow–Swan fundamental differential equation

**DOI:** 10.1016/j.heliyon.2022.e10816

**Published:** 2022-09-29

**Authors:** Norbert Brunner, Georg Mayrpeter, Manfred Kühleitner

**Affiliations:** Institute of Mathematics, Department of Integrative Biology and Biodiversity Research, University of Natural Resources and Life Sciences, Vienna, Austria

**Keywords:** Akaike information criterion (*AIC*), R-squared (*R*^2^), Simulated annealing, Solow–Swan growth model, Sum of squared errors (*SSE*), von Bertalanffy growth model

## Abstract

**Background:**

The Solow–Swan model describes the long-term growth of the capital to labor ratio by the fundamental differential equation of Solow–Swan theory. In conventional approaches, this equation was fitted to data using additional information, such as the rates of population growth, capital depreciation, or saving. However, this was not the best possible fit.

**Objectives:**

Using the method of least squares, what is the best possible fit of the fundamental equation to the time-series of the capital to labor ratios? Are the best-fit parameters economically sound?

**Method:**

For the data, we used the Penn-World Table in its 2021 version and compared six countries and three definitions of the capital to labor ratio. For optimization, we used a custom-made variant of the method of simulated annealing. We also compared different optimization methods and calibrations.

**Results:**

When comparing different methods of optimization, our custom-made tool provided reliable parameter estimates. In terms of R-squared they improved upon the parameter estimates of the conventional approach. Except for the USA, the best-fit values of the exponent were unplausible, as they suggested a too large elasticity of output. However, using a different calibration resulted in more plausible values of the best-fit exponent also for France and Pakistan, but not for Argentina and Japan.

**Conclusion:**

Our results have shown a discrepancy between the best-fit parameters obtained from optimization and the parameter values that are deemed plausible in economy. We propose a research program to resolve this issue by investigating if suitable calibrations may generate economically plausible best-fit parameter values.

## 1 Introduction

### 1.1 Goal of the paper

The fundamental differential Eq. (1) of the Solow (1956) and Swan (1956) model of capital accumulation aims at describing the capital (*K*) to labor (*L*) ratio, *k* = *K*/*L*, as a function of time, *t* (Barrow and Sala-i-Martin, 2004):

(1) $$\frac{dk\left(t\right)}{dt}=p\cdot k{\left(t\right)}^{a}-q\cdot k\left(t\right)$$

Eq. (1) has four parameters: exponent, *a*, scaling parameters, *p* and *q*, and the initial value, *k*(*t*_0_) = *k*_0_ at initial time *t*_0_. This paper asks: Given a time-series of observed values of capital to labor ratios, *k*_*i*_ at time *t*_*i*_ (*i* = 1, …, *N*), what are the best-fit parameters of the Solow–Swan differential equation, using the method of least squares? Thereby, we interpret Eq. (1) as an “empirical model” (Yue and Ducharme, 2016): We focus on data-fitting and ignore the economic interpretation of the parameters. As noted by Klemp (2013), this research question has rarely been discussed (c.f. Khoo et al., 2021).

The article "Parameter estimation of the Solow–Swan fundamental differential equation" was published in 2022. Journal: Heliyon.

This approach differs from the conventional “mechanistic modeling” that is common in undergraduate teaching, where the parameters are chosen from other data sources according to their economic meaning. (This is explained in Table 1 below.) Moreover, we ask if in hindsight the values of the best-fit parameters are economically meaningful.

**Table 1:** Derivation and economic interpretation of Eq. (1) in terms of the Solow–Swan model.

*key phrase*	*Formula*	explanation
initial variables	*Y*, *K*, *L*, *I*	output, capital stock, labor, investment
Cobb-Douglas equation:	$Y=A\cdot K^{\alpha }\cdot L^{1-\alpha }$	A productivity factor, *α* elasticity of output
investment = savings:	I=s⋅Y	*s* savings rate
capital accumulation with depreciation:	$\frac{dK}{dt}=I-d\cdot K=s\cdot A\cdot K^{\alpha }\cdot L^{1-\alpha }-d\cdot K$	*d* rate of depreciation of capital
Malthusian law:	$\frac{dL}{dt}=n\cdot L$	*n* exponential growth rate
quotient rule of calculus:	$\frac{d\left(\frac{K}{L}\right)}{dt}=\frac{\left(\frac{dK}{dt}\right)}{L}-K\cdot \frac{\left(\frac{dL}{dt}\right)}{L^{2}}$	*K*/*L* = *k*, capital per labor
substitute above equations:	$\frac{d\left(\frac{K}{L}\right)}{dt}=\frac{\left(s\cdot A\cdot K^{\alpha }\cdot L^{1-\alpha }-d\cdot K\right)}{L}-K\cdot \frac{\left(n\cdot L\right)}{L^{2}}$	
fundamental differential equation:	$\frac{dk}{dt}=s\cdot A\cdot k^{\alpha }-d\cdot k-n\cdot k$	simplify, using *k* = *K*/*L*
	$\frac{dk}{dt}=p\cdot k^{a}-q\cdot k$	simplify, using *a* = *α*, *p* = *s*·*A*, *q* = *d* + *n*
initial value	*k*(*t*_0_) = *k*_0_	*t*_0_, *k*_0_ > 0
steady state (equilibrium)	$k_{equ}=\sqrt[{1-a}]{p/q}$	solve *p k*^*a*^−*q k* = 0 = limit of *k*(*t*) for *t*→*∞*
analytic solution	$k\left(t\right)=k_{equ}\cdot \sqrt[{1-a}]{1-\left(1-{\left(\frac{k_{0}}{k_{equ}}\right)}^{1-a}\right)\cdot e^{-p\cdot \left(1-a\right)\cdot \left(t-t_{0}\right)/{\left(k_{equ}\right)}^{1-a}}}$	

***Note****:* Adapted from Acemoglu (2013), using common economic notation.

### 1.2 Background on teaching

The “Solow–Swan model” has been a milestone towards the development of modern growth theory (Chu, 2018) and it is still an active research topic (Google Scholar: 1800 publications since 2015 mentioning it). It is therefore included in most undergraduate curricula for economics (Ogun, 2014). In class, it was used to teach students the work with macroeconomic data (Wuthisatian and Thanetsunthorn, 2019) and to expose them to research experiences (example: Bellew, 2011; Frey, 2017).

The article "Parameter estimation of the Solow–Swan fundamental differential equation" was published in 2022. Journal: Heliyon.

Undergraduate teaching (Mixon and Sockwell, 2007; Stein, 2007; Jones and Vollrath, 2013) generally interpreted Eq. (1) as part of a larger “mechanistic model” describing the long-term growth of a country’s economy using merely two explanatory variables, labor and capital, ignoring (at first) distinctions within labor and capital. When the Solow–Swan model was fitted to data, then the economic parameters mentioned in the model equations of Table 1 were used. (Their values were outcomes of other lines of research, such as Hall, 1971; Hulten and Wykoff, 1981; Nadiri and Prucha, 1996 for depreciation.) Teaching then focused on comparisons of countries, often assuming the steady state (*k*_*equ*_ in Table 1) and linear models (as in research: Durlauf et al., 2005). The research question of this paper asks to abstract from the economic reasoning and consider Eq. (1) in isolation: We fit (1) to the data *k* = *K*/*L*, ignoring any other data and the meaning of the parameters.

### 1.3 Related economic growth models

The Solow–Swan model was adapted to take care of (exponentially increasing) technological progress. In this case, Eq. (1) holds for the capital to “effective labor” ratio (section 14 in Solow, 1956). Related adaptions allowed to discuss interdisciplinary issues in class, such as climate change (Tsigaris and Wood, 2016), corruption (Elmslie and Tebaldi, 2010), education (Breton, 2013), or over-exploitation of natural resources (Van den Berg, 2012). As our data do not inform about effective labor directly, this paper does not consider these adaptions.

Further, as our paper focuses on the fundamental equation of the Solow–Swan theory, we do not consider the modern approaches to economic growth theory, such as the Ramsey-Cass-Koopmans model, which endogenizes the savings rate (c.f. the outline in Spear and Young, 2014), or the Mankiw–Romer–Weil model, which extends the classical model by augmenting the production function with human capital (Mankiw et al., 1992). The differential equations of these and related models are summarized in Tsoularis (2021).

The fundamental Eq. (1) was modified by more realistic assumptions about the growth of labor, such as logistic growth (Mingari Scarpello and Ritelli, 2003), Richard’s growth (Accinelli and Brida, 2005), von Bertalanffy growth (Guerrini, 2010), general bounded growth (Guerrini, 2006; Ferrara, 2011a), or even decay (Ferrara, 2011b). However, this leads to different differential equations (and to difference-differential equations: Cai, 2012), which we do not consider here.

The article "Parameter estimation of the Solow–Swan fundamental differential equation" was published in 2022. Journal: Heliyon.

Moreover, this paper does not consider Eq. (1) with the exponent *a* = 1, as in the limit *a*→1^−^ (from below) differential Eq. (1) converges to the (different) Gompertz equation (Marusic and Bajzer, 1993). Yet, we consider *a* = 0, as Eq. (1) remains meaningful with this exponent (though elasticity *α* = 0 may not be realistic, economically).

Differential Eq. (1) remains meaningful for *q* = 0. In this case, the analytic solution is a power function with an infinite steady state. However, except for an example, in this paper we assume *q* > 0, as an infinite steady state would be incompatible with the *raison d’être* of the Solow–Swan model, namely the prediction of growth to a finite steady state, whose size can be controlled by growth policies (Solow, 1988).

### 1.4 Link to mathematical biology

The pros and cons of the empirical approach and of the above mechanistic approach towards Eq. (1) can be explained with reference to mathematical biology. There, Eq. (1) has been derived from a mechanistic biophysical model for the growth of animals, the generalized “von Bertalanffy model”, which is an active research topic, too (Google Scholar: 2300 publications since 2015 mentioning this term). In biological growth models, *k* means body mass and its growth is determined from the antagonistic effects of anabolism and catabolism, whereby the body utilizes resources at a metabolic rate for growth, the term *p*·*k*^*a*^, except for the resources allocated to the operation and maintenance of existing tissue, which are proportional to mass, the term *q*·*k* (Pütter, 1920).

By refining this reasoning, Bertalanffy (1957) argued that vertebrates would grow according to model (1) with the metabolic exponent *a* = 2/3. West et al. (2001) contested this claim and proposed the exponent *a* = 3/4. To resolve this controversy (Isaac and Carbone, 2010), biologists turned to the empirical modeling approach: They sought the best-fit exponents of Eq. (1) for distinct species and for different individual animals of the same species. It turned out that model (1) was not sufficient and a generalization with two exponents (*a*, *b*) was needed to accurately describe certain size-at-age data (Pauly and Cheung, 2018). For example, in a study of nestlings of blue tits from an urban park, each bird had its own optimal exponent (pair) that was unrelated to the metabolic exponents proposed by Bertalanffy and West. Rather, the model parameters were associated to small variations in the environment around each nest site (Brunner et al., 2021), whence the exponents were no longer interpreted in terms of metabolism. Instead, they were related to the shape of the size-at-age data (specifically to the ratio of the size at fastest growth over adult size).

The article "Parameter estimation of the Solow–Swan fundamental differential equation" was published in 2022. Journal: Heliyon.

Returning to the Solow–Swan model, we argue that an empirical approach may supplement the mechanistic modeling in the same way: When the best-fit parameters deviate from the parameters expected from the mechanist reasoning, this may indicate economic causes that future research might uncover.

## 2 Materials and method

### 2.1 Materials

We used Mathematica 13.0 (Wolfram Research, 2021) for computations. For economics courses that use Python (Jenkins, 2022), similar functions are available in Python libraries.

### 2.2 Data

We used PWT (2021), the 2021 Penn World Table, as in economic growth theory this is a well-established source of data collected annually from 1950 to 2019 (Feenstra et al., 2015). Thus, outside of China and Italy (which we do not consider) data were not affected by the Covid-19 pandemics.

First, we compared the fit of model (1) to the data from 1950 to 2019, using different definitions of the ratio, *k*, for the USA. For the capital stock, *K*, we used the variable cn (column “capital stock in million US dollars of 2017 at current purchasing power parities”), and for labor, *L*, we used the variable emp (“number of persons engaged in millions”). This resulted in the time series *k* = cn/emp.

Further, we considered, for *K*, the variable rnna (column “capital stock at constant 2017 national prices in million US dollar of 2017”), and defined the ratio *k* = rnna/emp. It differed only slightly from cn/emp, but we wished to explore by an example, if slight differences in the data would affect the growth curves.

For labor, *L*, we also considered another variable kh (“annual performed working hours in 1000 h”). We computed it from the variables emp and avh (“average annual hours worked by persons engaged”) as kh = emp × avh/1000. Using it, we defined the time series *k* = cn/kh.

In addition, we checked, if another macro-economic time series with a different meaning may be described well by Eq. (1). Using the variable ccon (“real consumption of households and government, at current purchasing power parities in million US dollars of 2017”) and the variable pop (column “population in millions”), we considered the time series *k* = ccon/pop. Note that ccon/pop is unrelated to capital per labor; it is also unrelated to per capita GDP. This time series displayed a steeper growth (ratio 4.16 of the 2019 value over the 1950 value) than cn/kh (ratio 2.92), and cn/emp (ratio 2.59).

The article "Parameter estimation of the Solow–Swan fundamental differential equation" was published in 2022. Journal: Heliyon.

Further, starting from cn/emp, we explored how to change the data to improve the fit. We considered “cn/emp modified”, where we removed a hypothesized trend, and “cn/emp aggregated”, where we smoothened the data using mean values.

Subsequently, we fitted Eq. (1) to the capital to labor ratios, *k* = cn/emp for the years 1950–2019, for a random sample of six countries. We did not consider countries, where data for cn or emp were missing. Further, with one exception (DR Congo), we disregarded countries, where a plot of *k* indicated no growth. The considered countries were Argentina, DR Congo, France, Japan, Pakistan, and USA. For the USA, we also considered the subset of the data from 1970 to 2009. This was an arbitrary choice, as we wished to check if the exponent would remain stable for sub-periods.

### 2.3 Calibration

To fit (1) to given data, we did not use the parametrization of the analytic solution in Table 1 (exponent *a*, scaling parameter *p*, initial value *k*_0_, and steady state *k*_*equ*_), but we solved differential Eq. (1) numerically (with current software no notable loss in precision). Hence, the four parameters *a*, *p*, *q*, and *k*_0_ were optimized (using *t*_0_ = *t*_1_ of the first data point).

We used the method of least squares, which seeks parameters of differential Eq. (1) that for the solution, *k*(*t*), minimize the sum of squared errors, *SSE* of Eq. (2). *N* is the count of the data (*N* = 70 for most of our data) and *k*_*i*_ are the data at time *t*_*i*_. *SSE*_*min*_ is the least *SSE*. If the value, *a*, of the exponent was given, then we defined *SSE*(*a*) as the least *SSE*, when three optimal parameters (*k*_0_, *p*, *q*) were sought for. For the best-fit exponent *a*_*min*_, *SSE*_*min*_ = *SSE*(*a*_*min*_).

(2) $$SSE=\overset{N}{\underset{i=1}{\sum }}{\left(k_{i}-k\left(t_{i}\right)\right)}^{2}$$

We considered another calibration, too: *SSLE*. To define *SSLE*, in Eq. (2) *k*_*i*_ is replaced by ln(*k*_*i*_) and *k*(*t*_*i*_) is replaced by ln(*k*(*t*_*i*_)). *SSLE* is less sensitive to heteroscedasticity (Kühleitner et al., 2019).

### 2.4 Optimization

For the minimization of *SSE*, we proceeded as follows: In the first step, we optimized *SSE*(*a*) for *a* = 0, 0.1, 0.2, ..., and 0.9 (step size 0.1) and identified *a*_1_ with the least *SSE*-value. In the second step, we repeated this in the interval between *a*_1_–0.1 and *a*_1_+0.1 (using step size 0.01). The optimization of each *SSE*(*a*) was based on simulated annealing (Vidal, 1993), using 50,000 simulated annealing steps. Simulated annealing uses a random search strategy to overcome the computational complexity of potentially NP-hard nonlinear global optimization problems (Horst and Pardalos, 2013; Pardalos and Vavasis, 1991): It chooses in each step random parameters from a neighborhood of the previous step, whereby, other than a random search, with a certain probability it also accepts suboptimal parameters and proceeds with them. (This allows the algorithm to escape from globally suboptimal local optima.) To finally focus on a promising parameter region, we let the diameters of the above-mentioned neighborhoods shrink by 5% after each 2500 steps. We thereby adapted the approach from Renner-Martin et al. (2018b). It allowed to detect problems with optimization if neighboring exponents displayed high fluctuations in *SSE*(*a*).

The article "Parameter estimation of the Solow–Swan fundamental differential equation" was published in 2022. Journal: Heliyon.

For verification of our custom-made optimization tool, we compared it with general-purpose methods of Mathematica: Levenberg-Marquardt method, which is common in nonlinear regression (Dennis and Schnabel, 1963), an interior point method (Potra and Wright, 2000), a differential evolution algorithm (Price et al., 2005), and the Nelder and Mead (1965) downhill simplex method. To ensure positive parameter values, in (1) we replaced parameter *p* by exp(*p*_*in*_ + *p*_1_) for some initial value (e.g., *p*_*in*_ = 0) and optimized for *p*_1_; the same for *q* and *k*_0_. We used these methods, as implemented in Mathematica, to fit model (1) with exponents *a* = 0, 0.1, ..., 0.9 to the data *k* = cn/emp of the USA and we compared *SSE*(*a*) and CPU time with the outcomes of simulated annealing. Further, we used them to compute, for a given best-fit exponent, 95% confidence intervals for the parameters *k*_0_, *p*, and *q*.

For a much simpler approach towards data-fitting, biologists used approximations to find parameters that may be close to the best-fit parameters. A common strategy (Kingdom and Azagba, 2017; Espino-Barr et al., 2015) is the Walford (1946) plot of *k′* over *k* (phase diagram), using numerical derivatives for *k′* (e.g.: *k′*(*t*) = *k*_*t*+1_ − *k*_*t*_ for *t* = *t*_0_, *t*_0_ + 1, ...). If the exponent, *a*, is given, then data-fitting in the phase diagram reduces to a linear regression, where parameters (*p*, *q*) are sought, so that the curve *f*(*k*) = *p*·*k*^*a*^ − *q*·*k* fits to the numerical derivatives, *k′*. With our data, this approach was not helpful. Another approach from animal science uses the Bertalanffy-Beverton plot (Renner-Martin et al., 2018a). However, to be feasible, this approach requires a-priori bounds for the steady state *k*_*equ*_ (in animal science: adult mass). Moreover, both methods apply for *SSE*, only.

### 2.5 Goodness of fit

In econometry, R-squared seems to be the most common statistics to assess the goodness of fit. As was noted by Mankiw (1997): *“I have always found the high R*^*2*^ *reassuring when I teach the Solow growth model.”* Thereby, in economic literature *R*^2^ > 0.9 is deemed a good fit. We therefore report *R*^2^, defined by Eq. (3). *RL*(*a*) is defined by replacing in this equation *SSE* with *SSLE* and *k*_*i*_ with ln(*k*_*i*_).

(3) $$R{\left(a\right)}^{2}=1-\frac{SSE\left(a\right)}{\sum_{i=1}^{N}{\left(k_{i}-mean\left(k_{1},k_{2},\ldots k_{N}\right)\right)}^{2}}$$

In view of criticism on R-squared (Achen, 1982), econometrists developed alternative definitions (e.g., Cameron and Windmeijer, 1997).

The article "Parameter estimation of the Solow–Swan fundamental differential equation" was published in 2022. Journal: Heliyon.

As was pointed out by Spiess and Neumeyer (2010), in nonlinear regression a high value of *R*^2^ may not be sufficient to select a true model, whereas the Akaike (1974) information criterion, *AIC*, would be much more selective. Eq. (4) defines *AIC* from *SSE* (Burnham and Anderson, 2002). In Eq. (4), *N* is the count of data and *K* is the number of optimized parameters. The model with a lower *AIC* is more parsimonious (more likely to be true).

(4) $$AIC\left(a\right)=N\cdot \text{ln}\left(\frac{SSE\left(a\right)}{N}\right)+2\cdot K$$

Following Renner-Martin et al. (2018b), we count *k*_0_, *p*, *q* and *SSE* as optimized parameters, but not the best-fit exponent, *a*_*min*_, because we identified it from a comparison of a small finite set of 29 growth models defined by different exponents. We also considered the fit to the model with *q* = 0; here we did not count the given *q* as a parameter.

(5) $$\text{prob}\left(a\right)=\frac{e^{-\Delta /2}}{1+e^{-\Delta /2}}\;\text{whereby}\;\Delta =AIC\left(a\right)-AIC_{min}$$

The Akaike weight, prob(*a*) of Eq. (5), is the probability that the best fit model with exponent *a* is true, when compared to the most parsimonious model, which by its definition has the least *AIC* = *AIC*_*min*_. If all models have the same number of parameters, this is the overall best fit model with exponent *a*_*min*_; *AIC*_*min*_ = *AIC*(*a*_*min*_). The Akaike weight assumes values between 0 and 0.5 (two models with equal fit and the same number of parameters each have 50% chance to be true). As above, we used *AIC* and prob also for *SSLE*, replacing *SSE* by *SSLE* in Eq. (4).

### 2.6 Statistics

The theory behind *SSE* assumes independent and identically normally distributed fit residuals (white noise); for *SSLE* a normal distribution of the corresponding differences of the logarithms is assumed. Under these assumptions, best-fit parameters from least squares are maximum likelihood estimations. This explains, why Eq. (4) could define *AIC* (originally defined by likelihood) in terms of *SSE*.

The article "Parameter estimation of the Solow–Swan fundamental differential equation" was published in 2022. Journal: Heliyon.

To verify these assumptions, we used the Cramér-von Mises distribution fit test (Xiao et al., 2006) and refuted the normal distribution hypothesis for P-values below 0.01, accepted it for P-values above 0.05, and interpreted values in between as “weak support” for that hypothesis. We also tested for significant autocorrelations, using the Box and Pierce (1970) test. In addition, we used an ACF-plot (autocorrelation function plot), showing the 95% confidence band and the correlations of the time-series of fit residuals with the lagged time series of residuals.

The variability of the parameters is higher than expected if the fit residuals are autocorrelated. First, the confidence intervals computed from the asymptotic normal distribution in parameter space are larger than estimated (Newey and West, 1987), because the derivation of the asymptotic distribution assumes independence of the errors. Second, the Akaike weights (4) assume independence of errors, too, whence their refutations of “false” models become dubious if this assumption is not satisfied. Nevertheless, we report confidence intervals and Akaike weights also in this case, but for a different purpose: Confidence intervals inform about the minimal expected variability of the best-fit parameters. And Akaike weights are used as a graphical method to detect problems with optimization (explained later in the text).

We did not compute confidence intervals for the best-fit exponents. This would require simulations, where the given data are perturbated by random errors. Then, for each simulation the optimization would be repeated. Neither did we study the stability of the parameters for different periods of time. Fisher (1921) suggested this as a criterion for model selection: If data follow e.g., the law of exponential growth, then the growth rate should be about the same, with smaller variations for larger sub-periods. (See Bhowmick et al., 2014, for generalizations.) This would require a parameter optimization for each sub-period of (at least four) consecutive years. Owing to the slow optimization, for both analyses the needed simulations were unfeasible.

## 3 Results

### 3.1 Best-fit parameters for USA data

Table 2 lists the best-fit parameters of Eq. (1), 95%-confidence intervals for *k*_0_, *p*, and *q* at the indicated best-fit exponent, and the goodness of fit for different definitions of the ratio, *k*, for the USA. Figure 1, Figure 2 summarizes the goodness of fit. Figures 2a and 3f plot the data, *k* = cn/emp, together with three different best-fit curves. Figure 3a plots fit residuals (Figure 4, Figure 5).

The article "Parameter estimation of the Solow–Swan fundamental differential equation" was published in 2022. Journal: Heliyon.

**Table 2:** Summary of the optimizations for the USA.

Data for the USA (definition of *k*, time span)		Best-fit parameters^a,b^ for model (1)				*k*_*equ*_	Goodness of fit	
		a	*k*_0_	p	q		SSE	*R*^2^
cn/emp, 1950–2019		0.37	1.73 × 10^5^	38.2	2.25 × 10^−6^	3 × 10^11^	5.39 × 10^9^	0.9887
confidence limit at *a* = 0.37	lower	0.37	1.68 × 10^5^	27.4	0^+^	NA		
	upper		1.79 × 10^5^	53.1	>10^10^			
cn/emp, 1950–2019, *q* = 0		0.37	1.73 × 10^5^	38.2	0	*∞*	5.39 × 10^9^	0.9887
confidence limit at *a* = 0.37	lower	0.37	1.69 × 10^5^	37.2	0	NA		
	upper		1.77 × 10^5^	39.2				
cn/emp modified^**c**^		0.32	1.75 × 10^5^	69.9	3.9 × 10^−5^	1.6×10^9^	1.58×10^9^	0.9965
confidence limit at *a* = 0.32	lower	0.32	1.71 × 10^5^	58.1	0^+^	NA		
	upper		1.78 × 10^5^	84.1	>10^10^			
cn/emp aggregated^d^		0.39	1.80 × 10^5^	29.7	1.5 × 10^−5^	2.1 × 10^10^	8.29 × 10^8^	0.9912
confidence limit at *a* = 0.39	lower	0.39	1.69 × 10^5^	17.4	0^+^	NA		
	upper		1.89 × 10^5^	63.6	0.83			
short-cn/emp, 1970–2009		0.99	2.48 × 10^5^	0.015	2.5 × 10^−4^	1.5 × 10^178^	1.95 × 10^9^	0.9785
confidence limit at *a* = 0.99	lower	0.99	2.44 × 10^5^	0.014	0^+^	NA		
	upper		2.52 × 10^5^	0.017	44 × 10^−4^			
cn/kh, 1950–2019		0.23	8.46 × 10^4^	157.9	2.4 × 10^−10^	2.3 × 10^15^	2.8 × 10^9^	0.9846
confidence limit at *a* = 0.23	lower	0.23	8.19 × 10^4^	148.8	0^+^	NA		
	upper		8.75 × 10^4^	167.5	>10^10^			
rnna/emp, 1950–2019		0.38	1.73 × 10^5^	33.62	1.1 × 10^−6^	1 × 10^12^	5.39 × 10^9^	0.9887
confidence limit at *a* = 0.38	lower	0.38	1.65 × 10^5^	28.04	0^+^	NA		
	upper		1.77 × 10^5^	54.74	0.02			
ccon/pop, 1950–2019		0.99	1.13 × 10^4^	1.06	0.93	2.7 × 10^5^	7.35 × 10^7^	0.9927
confidence limit at *a* = 0.99	lower	0.99	1.08 × 10^4^	0.847	0.74	NA		
	upper		1.18 × 10^4^	1.323	1.17			

*Notes*: ^**a**^) numbers rounded to the last shown decimal; ^**b**^) confidence limit 0^+^ for *q* means less than 10^−4^; ^**c**^) modified means cn/emp minus a hypothesized business cycle (Figure 4a); ^**d**^) aggregated means averages of cn/emp over successive five-year periods (Figure 2a). Computations using Mathematica 13.0.

**Figure 1:** Different evaluations for the goodness of fit of the best-fit solution of Eq. (1) with given exponent, *a*, for the USA data of Table 2 (legend in 1a); a) left: R-squared at *a*; b) right: Akaike weights at *a*. Computations using Mathematica 13.0 and plots using MS Excel & MS Power Point.

**Figure 2:** Plot of a) left: original data cn/emp (black), aggregated data (red: averages of successive five-year periods), and best-fit curve to the aggregated data (green); b) right: ACF plot of the fit residuals for the aggregated data (5 years lag between successive data points). Computations and plots using Mathematica 13.0.

The article "Parameter estimation of the Solow–Swan fundamental differential equation" was published in 2022. Journal: Heliyon.

**Figure 3:** Data (blue: cn/emp for 1950 to 2019) and best-fit model curves for *SSE* (red) and *SSLE* (green) for six countries: a) top left Argentina; b) top right DR Congo; c) middle left France; d) middle right Japan; e) bottom left Pakistan; and f) bottom right USA. Best-fit parameters are from Tables 4 and 5; plot using Mathematica 13.0.

**Figure 4:** Plot of a) left: fit residuals *r*_*i*_ = *k*_*i*_ − *k*(*t*_*i*_) for the best-fit curve *k*(*t*) with *a* = 0.37 (Table 2) to *k* = cn/emp (black dots) and the function *bc*(*i*) = 5480 1.015^*i*^ cos(2.38 + 0.17 *i*); b) right (ACF-plot): 95% confidence limits (dashed lines), autocorrelations of the fit residuals *r*_*i*_ (red dots), and autocorrelations (blue dots) of the best-fit residuals to the data *k*_*i*_ − *bc*(*i*), based on *k* = cn/emp and *a* = 0.32. Computations and plots using Mathematica 13.0.

The overall-best fit in terms of *R*^2^ was achieved by a “modified cn/emp”, using the exponent *a* = 0.32. However, these data were altered to achieve a better fit by removing a hypothesized business cycle (see below). The next best fit was achieved for ccon/pop, using the exponent *a* = 0.99. However, ccon/pop was a different time series, not related to capital per labor. Rank three was achieved for the fit to the aggregated data. However, this was a fit to 14 data points (rather than to 70) that were smoothened by averaging (see below). At rank four followed cn/emp and rnna/emp, and at rank five cn/kh.

For all data, except for short-cn/emp and ccon/pop, the R-squared values did barely vary for different values of the exponent, and except for short-cn/emp, a peak was barely discernible (Figure 1a). The Akaike weights were more selective insofar, as for all curves the peaks were clearly distinguishable (Figure 1b). However, there was still a high variability: Except for short-cn/emp and ccon/pop, no exponent *a* between 0.2 and 0.9 was refuted as unlikely (probability to be true below 5%). It follows that a slight change in the best-fit exponent could be offset by suitable changes of the other parameters, *c*, *p*, and *q*, resulting in a nearly optimal fit in terms of R-squared and an accepted fit in terms of the Akaike weight.

We compared these optimization results with a simple fictional “classroom approach”; Table 1 explains the notation. Starting with data about the USA from 1950 to 2019 (PWT, 2021), we used the variables cn, emp, and cgdpo for capital stock, labor, and output (*K*, *L*, and *Y*), respectively. Fitting exponential growth to *L* resulted in the estimate *n* = 1.42% for the growth rate of the workforce. The average of the annual depreciation rates, variable “delta”, delivered the estimate *d* = 3.57% for the capital depreciation rate. The average of the gross investment rates, variable csh_i, was an estimate for the savings rate (Leon Arias, 2010), *s* = 24.5%. The elasticity of output was assumed, *α* = 0.32 (optimal value). The productivity factor, *A* = 1373.1, was estimated from ln(*A*) = average of ln(*Y*/*L*)–*α*·ln(*K*/*L*); c.f. Cobb-Douglas equation. (Literature recommended a regression to obtain *α* and *A* simultaneously: Boyko et al., 2020.) This in turn provided the parameter estimates *p* = *A*·*s* = 336.6, *q* = *d* + *n* = 0.05, and *k*_*equ*_ = 4.3·10^5^. Using the initial value *k*_0_ = 168,386 at *t*_0_ = 1950 (first data points) defined a solution of (1) with *R*^2^ = 0.85.

The article "Parameter estimation of the Solow–Swan fundamental differential equation" was published in 2022. Journal: Heliyon.

These parameters did not achieve the best possible fit for cn/emp. However, an optimization of the exponent and of the initial value was an obvious step that could be done in a spreadsheet. (We used MS Excel and the Solver Add-In. Note that another value of *α* = *a* automatically altered the above estimates for *A*, *p*, and *k*_*equ*_.) It resulted in a significant improvement of the fit, *R*^2^ = 0.9861 (using *a* = 0.83). This was comparable to the best fit (*R*^2^ = 0.9887). In the same way, for rnna/emp *R*^2^ = 0.9884 (using *a* = 0.879) was close to the best fit (*R*^2^ = 0.9887), and for kh/emp *R*^2^ = 0.9068 (using *a* = 0.32) was more remote from the best fit (*R*^2^ = 0.9846). However, this approach failed for ccon/pop (it was a different time series, where the used economic parameters might not matter) and for short-cn/emp; the best fit was worse than the fit of the constant function “average of the data”.

### 3.2 Reliability of optimization

Our tool for finding the best-fit parameters was slow but practicable (ca. 45 minutes of CPU time per time-series on a standard business computer). By comparison, standard tools of optimization often resulted in parameter estimates with poorly fitting model curves (numerical instability), as was observed previously in mathematical biology (Loibel et al., 2010; Shi et al., 2014). Nevertheless, we used these standard methods to check, if they could improve the optimization of the parameters *k*_0_, *p*, and *q*, starting with the best-fit parameter values from our tool, and to compute their 95% confidence intervals (results in Table 2).

First, we used the plot of the Akaike weights (Figure 1b) to detect potential problems with optimization: For ccon/pop, the zig-zag lines in the plot of the Akaike-weights for *a* > 0.8 (Figure 1b) indicate that our simulated annealing tool did not always identify the least *SSE*(*a*) exactly. However, these fluctuations remained relatively small. The other curves had a smooth appearance.

The article "Parameter estimation of the Solow–Swan fundamental differential equation" was published in 2022. Journal: Heliyon.

Next, to verify our customized tool, we compared various methods of numerical optimization for *k* = cn/emp of the USA at ten test cases (optimization of *k*_0_, *p*, and *q* for the exponent *a* = 0, 0.1, ..., 0.9). The Levenberg-Marquardt method was ten times faster than our tool. It reduced *SSE* slightly in two test cases (meaning a reduction by at most 0.07%) and failed clearly in five cases (*SSE* by 10% higher). An interior point method was three times faster than our tool if we assumed *q* = 0. (Otherwise, it was much slower, but converged to *q* = 0, again.) It reduced *SSE* slightly in four test cases, but it failed clearly in three cases. The Nelder-Mead method needed three times the CPU time of our tool, improved *SSE* slightly in six test cases and failed clearly in two cases. Differential evolution needed nine times the CPU time of our tool, failed clearly in one test case and reduced *SSE* slightly for eight test cases. (We used *p*_*in*_ = 0; the same for the other parameters. Performances could be improved using a different *p*_*in*_ and by changing the default adjustments of the algorithms.) Summarizing, all methods confirmed the *SSE*(*a*) values of our tool, as they could improve them slightly at best. Thus, our custom-made simulated annealing tool provided reliable estimates for *SSE*(*a*), which was crucial for the identification of the best-fit exponent, and with an accuracy of ±10% these methods confirmed the best-fit values of the parameters *p* and *k*_0_.

The optimization of the parameter *q* (and therefore also of the steady state) was problematic, as is illustrated by a comparison of the almost equal data cn/emp and rnna/emp, but different steady states. The fluctuations of the steady states at different values of the exponent (Figure 5a) suggested a random pattern. Indeed, the optimization by means of simulated annealing defined a random path towards the optimum that was trimmed after a fixed number of annealing steps (50,000), whence a different path might lead to a different output of optimization. The optimization of the parameter *q* was problematic for other optimization methods, too, resulting in large confidence intervals (Table 1). Moreover, different runs of the optimization (different random numbers) moved the estimates for *q* closer to *q* = 0. The reason for this behavior was our assumption *q* > 0: As *q* = 0 implies an infinite steady state, *k*_*equ*_ = *∞*, we designed the algorithms to guarantee *q* > 0 (using *q* = exp(*q*_1_) and optimizing for *q*_1_). Therefore, when the best fit was achieved at or very close to *q* = 0, then the algorithms might terminate somewhere else at random (on the path to *q*_1_ = −*∞).*

The article "Parameter estimation of the Solow–Swan fundamental differential equation" was published in 2022. Journal: Heliyon.

**Figure 5:** Comparisons of model curve characteristics for different data; a) left: ln(*k*_*equ*_(*a*)), logarithm of the steady state at given exponent *a* for the USA data of Table 2 (legend in Figure 1a), whereby values above 50 (short-cn/emp for *a* > 0.8) were not displayed; b) right: comparison of best-fit models to *k* = cn/emp with given exponent *a* and *q* > 0 (red) or *q* = 0 (blue) with the most parsimonious model (*a*_*min*_ = 0.37, *q* = 0) in terms of Akaike weights (left axis) and R-squared (right axis). Computations using Mathematica 13.0 and plots using MS Excel & MS Power Point.

This limitation of optimization could not be overcome by more refined methods, because the data did not allow to discern the steady state from a visual inspection. In animal science, estimates for the steady state that were not evident from the data (adult size) were refuted as speculative (Knight, 1968). Rather, in such a situation an empirical approach might postulate an infinite steady state (*q* = 0) for the capital to labor ratio. To explore this alterative model assumption, we repeated the optimization for *k* = cn/emp with *q* = 0. This resulted in the same best-fit exponent, *a*_*min*_ = 0.37, with about the same *SSE* (Table 1). Therefore, the growth model with *q* = 0 was more parsimonious than the model with *q* > 0 (lower *AIC*): Owing to the penalty for the additional optimized parameter (*q* > 0) in *AIC*, the probability that the best-fit model with *q* > 0 was true, when compared to the best fit model with *q* = 0, was only 27%. Further, for *q* = 0 the peaks of the R-squared and Akaike weight curves were more distinct (Figure 5b) and the confidence intervals for *k*_0_ and *p* were smaller.

We conclude that the problems related to the steady state were not failures of optimization, but rather the consequences of a misfit between the model assumption (*q* > 0) of a finite steady state and data suggesting growth ad infinitum. It could be remedied easily (accepting an infinite steady state using *q* = 0). In the “classroom approach”, *q* > 0 followed from data unrelated to the capital to labor ratio and this did hide the potential unboundedness of the growth function.

### 3.3 Improving the data

For the time-series *k* = cn/emp we scrutinized the implicit assumptions for the method of least squares. We noted a good fit of the data and of the best-fit residuals to a normal distribution (Table 3). However, the residuals displayed a periodic structure, resulting in significant autocorrelations. Significant autocorrelations were observed also for the best-fit residuals of the other data of this paper when the Solow–Swan model was fitted to them. Such a failure of the white noise assumption may indicate a misspecification of the model. A common recommendation is to use a different model. If this is not viable, as a specific model is already established, there is an extensive literature on altering the data to make them fit better to the model by removing significant autocorrelation (Google Scholar: ca. 9500 papers about “pre-whitening” since 2015). However, this pre-whitening may lead to incorrect assessments of the significance of a trend (Yue et al., 2002). This section illustrates two other approaches.

The article "Parameter estimation of the Solow–Swan fundamental differential equation" was published in 2022. Journal: Heliyon.

**Table 3:** Tests for the goodness of the fit of a normal distribution.

Country	Tests for *SSE*		Tests for *SSLE*	
	Data *k*_*i*_	Residuals *k*_*i*_ – *k*(*t*_*i*_)	Data ln(*k*_*i*_)	Residuals ln(*k*_*i*_) – ln(*k*(*t*_*i*_))
Argentina	<0.0001	0.0059	<0.0001	0.0012
DR Congo	0.0302	0.0902	0.2938	0.2027
France	<0.0001	0.0004	0.0044	0.0115
Japan	<0.0001	<0.0001	<0.0001	0.0304
Pakistan	<0.0001	0.0013	0.0141	0.6108
USA	0.0988	0.0864	0.2213	0.0136

*Note:* P-values of the Cramér & von Mises tests, if the data cn/emp or the fit residuals to the best fit curve (1) with respect to the calibrations *SSE* and *SSLE* were normally distributed. Computations using Mathematica 13.0.

To remove the autocorrelations, we hypothesized a slow business cycle *bc* with increasing amplitude (red line in Figure 4a; formula for *bc* in the figure caption). For, business cycles may push consecutive data *k*_*i*_ systematically away from their trend *k*(*t*), whereby during upswing/downswing years the capital per labor ratio presumably was a higher/lower than in the trend, whence in general the fit errors for consecutive years deviated into the same direction, resulting in autocorrelations. We removed the cycle from the data and fitted Eq. (1) to the resulting modified time series *k* = cn/emp − *bc*. We obtained the best-fit exponent *a* = 0.32 with the highest *R*^2^ amongst the considered USA data. Its fit residuals were smaller and normally distributed (distribution fit test: P-value 0.24). The autocorrelations (Figure 2b) were smaller, but still significant (though for fewer time lags), as was confirmed by the Box-Pierce test.

As an alternative approach we fitted model (1) to aggregate data, the averages of cn/emp over five-year periods (14 data points). Figure 5a plots the raw data, the aggregated data (these are not moving averages), and the model curve fitted to the aggregated data. The best-fit model (exponent *a* = 0.39) had normally distributed fit residuals (P-value 0.55). Figure 5b is the ACF plot for the fit residuals: As was confirmed by the Box-Pierce test, there were no significant autocorrelations (except the trivial one for lag 0), but the correlations were not small. The confidence intervals for the parameters were larger, too (Table 2), and the Akaike weights did not refute any exponent (Figure 1b). Still another approach (similar outcome) would be pruning (e.g., selecting every fifth data-point).

The article "Parameter estimation of the Solow–Swan fundamental differential equation" was published in 2022. Journal: Heliyon.

Both approaches had drawbacks: The hypothesized business cycle (estimated from the fit residuals) might be an artefact of data-fitting, as in literature we could not identify a documented cycle with a 37-year period (between a Kuznets swing and a Kondratiev wave). The use of aggregate data did not remove the autocorrelations, but it merely reduced their significance owing to the smaller sample size. We therefore followed another recommendation (Storch, 1999) to handle autocorrelations: We continued to work with the Solow–Swan model (as it was supported from a mechanistic reasoning) and we used the unaltered data, but we were careful with statements about the reliability of the outcomes, and we checked the plausibility of the model parameters.

### 3.4 Plausibility of the best-fit parameters

According to Table 1, the scaling parameter, *p* of Table 2, has the meaning of a product of a savings rate, *s*, and an unknown productivity factor *A*, whence the plausibility of *p* was not assessed. The optimized initial values of Table 2 (parameter *k*_0_) were plausible, as their deviations from the initial values (*k*_1_) of the considered time-series were comparable to the deviations of the best-fit curves, elsewhere.

Next, we considered the best-fit values of parameter *q*. We noted two problems. First, the values obtained from optimization were problematic (see above). And second, these values were not plausible, economically. Except for ccon/pop (a time series with a different meaning, where these considerations did not apply), the value of *q* was close to zero and thus too small. For, in Table 1, the parameter *q* was expected to relate to the much larger sum of the labor growth rate (about 1%) and the capital depreciation rate. (However, considering the 95%-confidence interval, plausible values for *q* were conceivable for *k* = cn/emp.)

Finally, we considered the best-fit exponent, *a* of Eq. (1). It is generally linked to the elasticity of output with respect to capital, *α* in Table 1. Economic literature deems values around *α* = 1/3 as plausible, as according to Kaldor (1957) this would be the share of national income that goes to capital. Mankiw et al. (1992) derived values between 0.36 and 0.6, using a broad definition of capital (physical and human capital, the latter not considered in this paper), and Munguia et al. (2019) arrived at time dependent values of elasticity between 0.5 and 0.75. Amongst the unaltered time-series from Table 2, the best-fit exponent for cn/emp, *a* = 0.37, was closest to the plausible value *α* = 1/3. Further, when the data were altered to obtain a better fit (modified and aggregated cn/emp), the best-fit exponents remained close to the plausible value *α* = 1/3. Therefore, this paper focused on cn/emp. For short-cn/emp, the best-fit exponent, *a* = 0.99, was not plausible economically. Further, for all time-series with *q* > 0, with probability 20% or higher, any economically unplausible exponent *a* ≥ 0.9 could be true.

The article "Parameter estimation of the Solow–Swan fundamental differential equation" was published in 2022. Journal: Heliyon.

### 3.5 Best-fit growth curves for various countries

To explore the situation for different countries, we fitted Eq. (1) to the capital to labor ratios for a random sample of countries; we used the ratios *k* = cn/emp and applied two calibrations, *SSE* and *SSLE*. The different calibrations resulted in different outcomes: Table 4 list the best-fit parameters for *SSE*, Table 5 is a list for *SSLE*, and Table 3 informs about the test results for the normal distribution assumptions inherent to these calibrations. Figure 3 plots the data and best-fit curves with respect to both calibrations. Figure 6 compares the Akaike weights with respect to *SSE* and *SSLE*.

**Table 4:** Optimization outcomes for *SSE* and selected countries.

Data (county)	Best-fit parameters for model (1)				*k*_*equ*_	Goodness of fit	
	a	*k*_0_	p	q		SSE	*R*^2^
Argentina	0.90	0.244	1.756	0.513	2.18 × 10^5^	2.3 × 10^10^	0.9140
DR Congo	0.98	4.2×10^3^	6.51	5.37	1.48 × 10^4^	7.1 × 10^8^	0.4347
France	0.99	9.87 × 10^4^	0.03	3.08 × 10^−5^	2.06 × 10^299^	1.2 ×10^11^	0.9309
Japan	0.97	1.58 × 10^3^	2.54	1.71	5.11 × 10^5^	5.6 × 10^10^	0.9651
Pakistan	0.91	3.12 × 10^3^	0.076	7.52 × 10^−4^	1.92 × 10^22^	1.2 × 10^8^	0.9721
USA short	0.99	2.48 × 10^5^	0.015	2.5 × 10^−4^	1.5×10^178^	1.95 × 10^9^	0.9785
USA	0.37	1.73 × 10^5^	38.2	2.25 × 10^−6^	3 × 10^11^	5.39 × 10^9^	0.9887

*Note:* Fit of model (1) to *k* = cn/emp for 1950 to 2019, using *SSE*. Numbers rounded to the last shown decimal; computations using Mathematica 13.0.

**Table 5:** Optimization outcomes for *SSLE* and selected countries.

Data (county)	Best-fit parameters for model (1)				*k*_*equ*_	Goodness of fit	
	a	*k*_0_	p	q		SSLE	*RL*^2^
Argentina	0.99	8.16 × 10^3^	0.14	0.08	1.65 × 10^25^	4.29	0.9511
DR Congo	0.97	4.83 × 10^3^	4.48	3.37	1.42 × 10^4^	3.89	0.5564
France	0.47	8.12 × 10^4^	19.24	3.27 × 10^−6^	5.93 × 10^12^	1.14	0.9517
Japan	0.99	1.35 × 10^4^	2.98	2.59	1.03 × 10^6^	1.82	0.9798
Pakistan	0.57	2.38 × 10^3^	1.75	1.37 × 10^−5^	7.57 × 10^11^	1.09	0.9715
USA short	0.99	2.50 × 10^5^	0.015	7.59 × 10^−4^	2.54 × 10^129^	0.017	0.9792
USA	0.16	1.69 × 10^5^	536.2	3.76 × 10^−7^	7.91 × 10^10^	0.052	0.9908

*Note:* Fit of model (1) to *k* = cn/emp for 1950 to 2019, using *SSLE*. USA short are the data from 1970 to 2009. Numbers rounded to the last shown decimal; computations using Mathematica 13.0.

The article "Parameter estimation of the Solow–Swan fundamental differential equation" was published in 2022. Journal: Heliyon.

**Figure 6:** Akaike weights for the best-fit solution of Eq. (1) for the time-series *k* = cn/emp for the five countries of Table 4 (legend in Figure 2a): a) left: prob(*a*) terms of *SSE*; b) right: prob(*a*) in terms of *SSLE*. Optimizations using Mathematica 13.0 and plot using MS Excel and Power Point.

Amongst the considered countries, the fit of model (1) to the data cn/emp was worst for the Democratic Republic of the Congo (*R*^2^ = 0.43, *RL*^2^ = 0.56). The best-fit model curves for *SSE* and *SSLE* (Figure 3b) were close together and followed the initial growth phase, but apparently, they were unrelated to the data, otherwise. This was also reflected by the indeterminateness in terms of the Akaike weights (Figure 6a): For *SSE* and *SSLE*, the best fit exponents were 0.98 and 0.97, respectively, but (except for prob(0.99) < 5% for *SSE*) all values for the exponent were likely to be true (30% or higher probability). Hence, growth modeling was futile and there was no discernible trend for growth. Indeed, DR Congo is amongst the poorest countries of the world, as since 1996 wars for its rich mineral resources and other conflicts led to mass starvation, displacements, and other severe social problems. The data indicate a demise already during the 1990s, the final phase of the Mobutu-regime.

For the Argentine Republic, the fit was reasonable (*R*^2^ = 0.91, *RL*^2^ = 0.95). There were large deviations of the data from the curve, as the best-fit model needed to accommodate three distinct phases: an initial sluggish slow growth of *k*, a steep rise starting during the 1980s (end of the military dictatorship and its dirty war in 1983), and high fluctuations with an overall slow growth since the 1990s (economic crisis 1999–2002). These deviations affected the two calibrations differently: For *SSE*, the best-fit curve started with an initial value close to 0 and it finally flattened to follow the final phase of slow growth. This flattening resulted in a S-shape. For *SSLE*, the best-fit curve started close to the initial data points and there was no discernible S-shape. For both growth curves the best fit exponents, 0.9 and 0.99, respectively, were economically unplausible. As for both calibrations the inherent normal distribution assumptions were refuted (Table 3), care was needed with an interpretation of the data-fitting. Further, for the calibration *SSE* we observed difficulties with the optimization, as there were high fluctuations (by 10% or more) of the Akaike weights close to the best-fit exponent. Notably, considering *SSE* and the best-fit exponent *a* = 0.9, the best-fit parameters were improved during the second round of optimizations; from *R*^2^ = 0.913 in the first round to *R*^2^ = 0.914. For *SSLE*, we did not observe a similar difficulty with optimization.

The article "Parameter estimation of the Solow–Swan fundamental differential equation" was published in 2022. Journal: Heliyon.

For the French Republic, the fit was reasonable (*R*^2^ = 0.93, *RL*^2^ = 0.95). The best fit curves for *SSE* and *SSLE* followed similar trajectories. Moreover, for both calibrations the plot of the Akaike weights showed smooth curves indicating no problems with optimization. The main deviation of the growth curves from the data occurred around the recession of 2000: Capital per labor started to decline in 1995 and to regain momentum in 2003. Thereby, the best-fit curve for *SSE* was more strongly affected by this final growth phase. The values of the best-fit exponents, 0.99 and 0.48 for *SSE* and *SSLE*, respectively, were distinct. The latter value for *SSLE* was more plausible, economically, and the distribution fit tests provided a weak support for *SSLE*. For, testing if the fit residuals for *SSLE* were normally distributed resulted in a P-value above 0.01. By contrast, both normal distribution assumptions related to *SSE* were refuted (P-values below 0.01).

For the State of Japan (Nippon-koku), the fit of model (1) was good (*R*^2^ = 0.97, *RL*^2^ = 0.98). However, on a visual inspection the data displayed distinct fluctuations around the best-fit growth curves. As for Argentina, the best-fit model curves for *SSE* and *SSLE* differed. The data display an economic stagnation since the collapse of an asset price bubble in 1991, which resulted in a S-shaped curve for *SSE*, while the curve for *SSLE* did not display a discernible S-shape. The best-fit exponents, 0.97 and 0.99 for *SSE* and *SSLE*, respectively, were unplausible, economically. While the normal distribution assumptions for *SSE* were refuted (Table 3), there was a weak support for *SSLE* (P-value above 0.03 for normally distributed fit residuals for *SSLE*). Further, for *SSE* but not for *SSLE*, there were problems with optimization, indicated by high fluctuations of the Akaike weights close to *a* = 1.

Amongst the considered countries, we observed the second best fit of model (1) to the data for the Islamic Republic of Pakistan (*R*^2^ = 0.97, *RL*^2^ = 0.97). The good fit of both model curves (only small fluctuations of the data) and the continuous growth of *k* since 1950 were insofar surprising, as Pakistan is a developing country with an extremely poor population and low human development index (HDI = 0.557 = rank 152 in the world, source: United Nations, 2020). For both calibrations, the best-fit growth curves followed similar growth trajectories, but the values of the best-fit exponent were distinct, 0.91 for *SSE* and 0.57 for *SSLE*. For *SSE*, the normal distribution assumptions were refuted (Table 3), while there was strong support for the assumption of normally distributed residuals for *SSLE*. Further, both plots of the Akaike weights showed smooth curves, indicating no problems with optimization.

The article "Parameter estimation of the Solow–Swan fundamental differential equation" was published in 2022. Journal: Heliyon.

The best fit of model (1) was achieved for the United States of America (*R*^2^ = 0.99, *RL*^2^ = 0.99). For both calibrations, the best-fit growth curves were almost overlapping, and the best-fit values of the exponents were economically plausible, 0.37 and 0.16 for *SSE* and *SSLE*, respectively. The distribution fit tests supported both calibrations (Table 3), whereby two tests supported *SSE*. The plots of the Akaike weights were smooth (Figure 6), whence there occurred no problems with optimization. Further (Table 2), two modifications of the data to generate fit-residuals with insignificant autocorrelations (removing a hypothesized business cycle; aggregation over successive five-year periods) resulted in comparable best-fit exponents for *SSE*. Thus, amongst the data considered in this paper, the data for the USA displayed an exceptional outcome with respect to *SSE*. However, for the data of a shorter period (1970–2009) we observed an unplausible best-fit exponent (*a* = 0.99).

We checked also the “classroom approach”, that used literature data for several parameters and optimized only the exponent and the initial value (section 3.1 for the USA). This approach failed for DR Congo (there was no growth), achieved poor fits for Pakistan (*R*^2^ close to 0) and Argentina (*R*^2^ = 0.40), an acceptable fit for Japan (*R*^2^ = 0.88, remote from the optimal *R*^2^ = 0.97) and a close to optimal fit for France (*R*^2^ = 0.91, optimal *R*^2^ = 0.93).

## 4 Discussion

Using the method of least squares, we compared five time-series for different definitions of the capital to labor ratio of the USA. The most plausible best-fit exponent was achieved for the time series *k* = cn/emp. For these data we compared several standard methods of optimization. These methods were not practicable (too slow or unreliable). Yet, taken together they confirmed the best-fit parameters *k*_0_ and *p* of our custom-made tool, and the best-fit estimate *SSE*(*a*), which was needed to optimize the exponent. However, the third parameter (*q*) was problematic, because we enforced the constraint *q* > 0, while for some data the “true” (least parsimonious) growth model would assume *q* = 0 with an infinite steady state, which would be implausible, economically. Further, for several data the fit residuals were not normally distributed and for all data there were significant autocorrelations for the fit residuals (comparable to Figure 5a). From plots of the residuals, we hypothesized that the data were disturbed by business cycles. For cn/emp of the USA, this hypothesis partially explained the autocorrelations.

The article "Parameter estimation of the Solow–Swan fundamental differential equation" was published in 2022. Journal: Heliyon.

Owing to the high variability, best fits were difficult to identify, but reasonable fits could be achieved for a wide range of parameters (defining a “reasonable fit” by *R*^2^ > 0.9); Figure 1a outlines this for the exponent. This explains, why the approach of undergraduate courses (Table 1) may have worked: Plugging in certain economic parameters into Eq. (1) and optimizing the exponent (elasticity) could result in reasonable fits (sections 1 and 3.1). By comparison, Akaike weights were more selective in assessing the goodness of fit: Other than for the rather flat curves of R-squared, for Akaike weights the peak around the best-fit exponent (*a*_*min*_) was clearly distinguishable. Nevertheless, also the variability of exponents that were not refuted by the Akaike weights was high.

We focused on the exponent and compared six countries, using cn/emp. Using *SSE* for calibration we could observe an economically plausible value for the USA, only. Using *SSLE* instead of *SSE* changed the picture somewhat and for three countries we obtained economically (more) plausible best-fit values for the exponent. This leads to the research question, if for some calibration economically meaningful best-fit parameters for the Solow–Swan fundamental equation can be extracted from empirical data. Are there a priori conditions on the data that ensure the success of this endeavor?

We conclude that the fundamental differential Eq. (1) is a suitable tool for analyzing the temporal evolution of the capital to labor ratio. Solow’s success story was a good motivation for this equation. However, the parameter values, which this story proposes, may not be exactly true and the best-fit parameters for Eq. (1) may not always be economically meaningful. We therefore suggest for the empirical approach that the exponent should not be equated with elasticity (*a* ≠ *α*). Rather, the exponent should be interpreted as a shape parameter of the time-series of the capital to labor ratios. A similar situation was observed in biology, where stories were told, why Eq. (1) and why certain exponents would be most suitable for explaining animal growth. However, when the model was fitted to growth data, environmental factors were more important than the proposed inherent metabolic mechanisms. We hypothesize by analogy with biology that for the Solow–Swan model, too, unknown or not yet modeled external factors may influence the shape of the growth data and thereby move the best-fit parameters, specifically the exponent, away from economically plausible values. The identification of such factors is proposed as another question for future research. Empirical analyses of the Ramsey-Cass-Koopmans and Mankiw-Romer-Weil models might be a starting point.

The article "Parameter estimation of the Solow–Swan fundamental differential equation" was published in 2022. Journal: Heliyon.

## Declarations

### Author contribution statement

Norbert Brunner, Manfred Kühleitner: conceived and designed the experiments; performed the experiments; analyzed and interpreted the data; contributed reagents, materials, analysis tools or data; wrote the paper.

Georg Mayrpeter: conceived and designed the experiments; analyzed and interpreted the data; contributed reagents, materials, analysis tools or data.

### Funding statement

This work was supported by Universität für Bodenkultur Wien.

### Data availability statement

Data associated with this study has been deposited at Reference PWT (2021) in the paper: Penn World Table 10.0, Link: www.ggdc.net/pwt.

### Declaration of interests statement

The authors declare no conflict of interest.

### Additional information

No additional information is available for this paper.
